# The Hydroalcoholic Extract of *Nasturtium officinale* Reduces Lung Inflammation and Oxidative Stress in an Ovalbumin-Induced Rat Model of Asthma

**DOI:** 10.1155/2022/5319237

**Published:** 2022-06-21

**Authors:** Nasrin shakerinasab, Mohammad Abbas Bejeshk, Hossein Pourghadamyari, Hamid Najafipour, Mahdieh Eftekhari, Javad Mottaghipisheh, Navid Omidifar, Mahdokht Azizi, Mohammad Amin Rajizadeh, Amir Hossein Doustimotlagh

**Affiliations:** ^1^Student Research Committee, Yasuj University of Medical Sciences, Yasuj, Iran; ^2^Physiology Research Center, Institute of Neuropharmacology, Kerman University of Medical Sciences, Kerman, Iran; ^3^Department of Physiology and Pharmacology, Afzalipour Medical Faculty, Kerman University of Medical Sciences, Kerman, Iran; ^4^Student Research Committee, Kerman University of Medical Sciences, Kerman, Iran; ^5^Department of Clinical Biochemistry, Afzalipour School of Medicine, Kerman University of Medical Sciences, Kerman, Iran; ^6^Department of Pharmacognosy and Pharmaceutical Biotechnology, Faculty of Pharmacy, Kermanshah University of Medical Sciences, Kermanshah, Iran; ^7^Center for Molecular Biosciences (CMBI), Institute of Pharmacy and Pharmacognosy, University of Innsbruck, Innrain 80–82, Innsbruck 6020, Austria; ^8^Biotechnology Research Center, Department of Pathology, School of Medicine, Shiraz University of Medical Sciences, Shiraz, Iran; ^9^Medicinal Plants Research Center, Yasuj University of Medical Sciences, Yasuj, Iran; ^10^Department of Clinical Biochemistry, Faculty of Medicine, Yasuj University of Medical Sciences, Yasuj, Iran

## Abstract

**Background:**

Asthma is known as a disease that causes breathing problems in children and adults and is also associated with chronic inflammation and oxidative stress of the airways. *Nasturtium officinale* (*NO*) possesses a wide range of pharmacological properties, particularly anti-inflammation and antioxidant potentials. Thus, this study for the first time was aimed to investigate anti-inflammatory and antioxidative activities of *NO* extract (*NOE*) in an ovalbumin-induced rat model of asthma.

**Materials and Methods:**

Forty-four male Wistar rats were sensitized with ovalbumin (OVA) to induce asthma symptoms. The animals were allocated into five groups: control (C), asthmatic (A), A + *NOE* (500 mg/kg), *NOE* (500 mg/kg), and A + dexamethasone (DX, 2.5 mg/kg). After 7 days, blood and tissue samples were taken from the rats. Then, the level of inflammatory markers, oxidative stress parameters, and antioxidant enzymes activity were measured.

**Results:**

The obtained results showed that OVA-sensitive rats significantly increased the levels of pro-inflammatory cytokines IL-1B, TGF-*β*, and SMA-*α* compared to the control group (*p* < 0.05), while treatment with *NOE* remarkably reduced the SMA-*α* gene expression compared to the asthma group (*p* < 0.05). Furthermore, it decreased the expression of IL-1B and TNF-*α* genes, although it was not statistically significant. The level of glutathione peroxidase (GPX) significantly reduced in *A* group compared to the *C* group (*p* < 0.05), whereas *NOE* administration significantly increased this marker (*p* < 0.05). Moreover, *NOE* attenuated inflammation and alveolar injury in the lungs of OVA-sensitive rat compared to the nontreated *A* group.

**Conclusions:**

Overall, our findings demonstrated that *NOE* somewhat is able to reduce airway inflammation by reducing inflammatory and increasing GPX activity. Indeed, further experiments investigating the impact of different extract doses are needed to confirm the antioxidant and anti-inflammatory effects of *NOE*.

## 1. Introduction

Asthma is a chronic respiratory disease with various clinical and pathophysiological profiles including increased mucus secretion, narrowing of the airways, reversible bronchial obstruction, goblet cell hyperplasia, airway hyper responsiveness (AHR), as well as identified acute and chronic inflammation [1, 2]. In addition to the aforementioned disease characteristics, asthma has recently been defined as a heterogeneous disease or complex syndrome and can be classified into several phenotypes and endotypes, each with specific clinical and pathological attributes [3, 4]. Asthma is one of the most common chronic diseases affecting children and adults worldwide [5, 6]. Currently, more than 315 million people in the world and approximately 12–14% of the Iran population suffer asthma; however, this rate concerningly increases by 50% every decade and puts a heavy burden on public health [7, 8]. In susceptible patients, the main asthma clinical symptoms consist of dry cough, breath shortness, wheezing, chest tightness, and even death [9]. The short-term and long-term corticosteroids and *β*-adrenergic agonists or leukotrienes are considered the therapeutic options for the treatment of asthma, although 5–10% of patients treated with them is failed [10].

Inflammation plays a key role in the pathophysiology of asthma. Inflammation of the airways is associated with the reaction of various immune cells and different mediators [11]. They secrete several immune cells, including *T* helper 2 cells (Th2), mast cells, eosinophils, airway epithelial cells, cytokines, chemokines, and inflammatory mediators that damage lung tissue [2]. Th2 lymphocytes produce cytokines such as interleukins-4, 5, and 13 (IL-4, IL-5, IL-13, respectively), leading to the production of immunoglobulin *E*, mucosal metaplasia, and increased production of eotaxins and eosinophils in the airways [9]. In addition, inflammatory epithelial cells produce high levels of pro-inflammatory cytokines and chemokines such as tumor necrosis factor *α* (TNF-*α*), interleukin-1*β* (IL-1*β*), and interleukin-6 (IL-6) [12, 13]. TNF-*α* acts as a neutrophil and eosinophil chemotaxis agent and increases the expression of epithelial cell adhesion molecules and is involved in organizing the airway inflammatory response [14]. IL-1*β* stimulates the production of Th2 after exposure to allergens, which in turn activates eosinophils at the site of airway inflammation and releases cytokines, including IL-5 [14]. IL-6 is an inflammatory cytokine possessing several functions including regulating bleeding, tissue regeneration, inducing chronic inflammation, maintaining autoimmunity, and tumorigenesis. IL-6 increases Th2 and enhances the effects of IL-4 and the survival of mast cells, thereby increasing airway responsiveness. Recent studies provide evidence that IL-6, rather than being involved in pneumonia, plays an important role in the pathogenesis of asthma [15].

Oxidative stress significantly involves in regulating inflammation as well as the pathogenesis of various chronic inflammatory diseases such as asthma [16, 17]. Asthma is associated with increased oxidative stress *via* activation of inflammatory cells such as monocytes, macrophages, neutrophils, and eosinophils which actively produce oxidant compounds such as reactive oxygen species (ROS) [18]. Oxidative stress occurs due to an imbalance between oxidant and antioxidant compounds. Oxidant compounds include ROSs (hydroxyl, superoxide, and hydrogen peroxide), reactive nitrogen species (RNS), and reactive sulfur species (RSS) [19]. Antioxidants are divided into two categories: enzymatic and nonenzymatic. The nonenzymatic antioxidants include vitamins A, C, and E, bilirubin, and glutathione, while the enzymatic ones comprise glutathione peroxidase (GPX), superoxide dismutase (SOD), and catalase (CAT); taking into account that the enzyme defense system is the first rapid line of defense against ROS [20, 21]. Total Thiol sulfhydryl (TSH) is an effective antioxidants that can preserve the correct structure of proteins, and can protect cells and tissues from damage induced by oxidative stress [22]. Free radicals can damage all macromolecules such as carbohydrates, proteins, lipids, and nucleic acids [19]. Thus, oxidative stress leads to hyperplasia of goblet cells and ultimately exacerbates inflammation by increasing the release of inflammatory cytokines and altering the function of antioxidant enzymes [23, 24].

Many studies have been conducted to demonstrate the beneficial therapeutic effects of herbal medicines, including antioxidant [25], anti-inflammatory [26], anticancer [27, 28], antimicrobial [29], and immune modulating effects [30–33]. *Nasturtium officinale* (*NO*) known as Watercress is a species of aquatic plant belonging to the cabbage family (Brassicaceae) that generally grows in cold, clear water [34]. *NO* contains vitamins A, B, C, E, folic acid, and high concentrations of glucosinolates as well as carotenoids such as *B* carotene, lutein, quercetin, and also contains some elements such as iodine, chromium, iron, calcium, and sulfur [35, 36].

The folk medicinal application of *NO* for the treatment of diabetes, bronchitis, diuresis, and influenza has been reported [34]. High antioxidant activity of the *NO* extract has been attributed to a variety of mechanisms and reactions, including inhibition of lipid peroxidation, prevention of hydrogen accumulation, and radical scavenging [37]. In addition to the high antioxidant effects, this plant exhibited to be potent as anti-inflammatory, antidiabetic, antiallergic, antibacterial, anticancer, and anticancer herbal remedy, possessing beneficial effects on the reproductive system [35, 38].

Considering the role of oxidants in asthma and airway inflammation and the antioxidant and anti-inflammatory effects of *NO* extract (*NOE*), the present study for the first time aimed to investigating the impact of NOE on oxidative and inflammatory stress markers in the rat model of ovalbumin-induced asthma.

## 2. Materials and Methods

### 2.1. Plant Material and Extraction

The stems and leaves of *NO* were collected in September 2020 from Kakan region located in Yasuj, Iran, and were identified by a botanist (Dr Jafari), while a voucher specimen (Herbarium no. HYU30230) was deposited in Yasuj University. They were cleaned after collection, and then shade dried, and powdered. About 100 g of the pulverized plant material was drenched with 1 L ethanol (70%, Yasan, Iran). The extraction was performed *via* maceration in incubator (37°C) for 48 h. After filtration, the filtrate was subsequently concentrated under a reduced pressure using a Rotavapor (Heidolph, Germany) at 40°C. The dried extract was stored in a refrigerator at ‒20°C until further experiments [39].

### 2.2. Animals

Male Wistar rats weighing 200–250 g (8–10 weeks old), purchased from the Animal Home of the School of Medicine, Yasuj University of Medical Sciences (Yasuj, Iran). The rats were kept under standard conditions of 12 h light/dark cycle, environment temperature of 22 ± 2°C, with free access to water and normal rodent chow. The study protocol was conducted according to “NIH US publication No. 86–23” for the care and use of laboratory animals and approved by the ethics committee of Yasuj University of Medical Sciences (Code: IR.YUMS.REC.1399.155).

### 2.3. Experimental Design

In the present study, 30 male Wistar rats accidentally were divided into five following groups: control group (*C*, *n* = 6), in which the normal saline was administered, asthmatic group (*A*, *n* = 6), where the rats were sensitized with OVA, asthma + *NOE* (*n* = 6) which were treated with 500 mg/kg *NOE* orally [34, 40] for a period of 7 days, only *NOE* (*n* = 6), asthma + dexamethasone (*A* + DTX, *n* = 5) rats which were received 2.5 mg/kg DTX intraperitoneally for 7 days.

Brieﬂy, in order to induce the allergic asthma model, rats were sensitized on days 0 and 7 by intraperitoneal injection of 1 mg ovalbumin (OVA) + 200 *µ*g aluminum hydroxide (Al(OH)_3_) in 0.5 mL phosphate buffered saline (PBS), and on days 14 to 42 of the protocol, they were challenged with inhaled OVA 1% using a nebulizer for 30 min every other day [14, 41]. At the end of day 50, the rats were anesthetized with an injection containing ketamine (80 mg/kg) and xylazine (10 mg/kg). The blood collected from animals was centrifuged to separate serum, and the serum samples were stored at −20°C for biochemical analysis. After sacrificing the rats, their lungs were removed and divided into two pieces. The first piece was stored in 10% formalin for histological examination, and the second piece was further kept at −70°C and utilized to study the gene expression [14]. For BALF collection, at the end of the experiment, median sternotomy was performed, the trachea was isolated, and the right main bronchus was clamped. A catheter was inserted to the left main bronchus of the animal and 2.5 mL of normal saline were instilled into the bronchoalveolar space of the left lung. The bronchoalveolar lavage fluid (BALF) was aspirated slowly after 5 min and centrifuged at 1500 g for 10 min at 4°C. The supernatant was removed and stored at −70°C oxidative stress markers analysis.

### 2.4. Measurement of Oxidants, Antioxidants, and Cytokines

#### 2.4.1. Determination of Oxidative Stress Tests

*(1). Determination of Antioxidant Enzymes Activity.* The activity levels of superoxide dismutase (SOD) and glutathione peroxidase (GPX) enzymes in lung tissue were evaluated based on the instructions of ELISA kit (ZellBio GmbH, Ulm, Germany) [7].

*(2). Determination of Cytokines.* Quantitative assessments of TNF-*α*, IL-6 and IL-10 was performed by Sandwich method with ELISA kit (Karmaia Pars gene Kerman, Iran), as previously described. The intra-assay CVs for IL-10, TNF-*α*, and IL-6 were less than 3%, and the interassay CVs for IL-6 and TNF-*α* were less than 8% and for the IL-10 was less than 9%. The lower limit of detection of IL-10 was 8 pg/mL, and that of TNF-*α* and IL-6 were 2 pg/mL.

### 2.5. RNA Isolation and Real-Time PCR

RNA was extracted from homogenized lung tissue by RNase Fibrous Tissue kit (Qiagen) based on manufacturer's protocol. Next, the complementary DNA (cDNA) was synthesized using a cDNA synthesis kit (Gene all, Korea). Finally, the expression of TNF-*α*, IL-1*β*, *α*-SMA, and IL-6 genes was determined using SYBR Green for quantitative real-time PCR. The difference in expression between the asthmatic and control mice related to the expression level of *β*-actin RNA was quantified using the 2^−ΔCt^ method [15].

### 2.6. Histological Examinations

For evaluation of changes at the histological stage, lung tissue sections were kept in 10% formalin. After dehydration in graded alcohol series, it was cleared in xylene. Then, the tissues were embedded in paraffin, sectioned and stained with haematoxylin and eosin reagent. The sections were studied by two observers, blind to the experimental groups [42].

### 2.7. Statistical Analysis

In this study, the obtained data were analyzed using one-way analysis of variance (ANOVA) following by Tukey's multiple comparisons. In all experiments, *p* values less than 0.05 was considered as significance level [43].

## 3. Results

### 3.1. Effects of *NOE* on Serum Oxidative Stress Markers

Data concerning serum oxidative stress markers (MDA, FRAP, TSH, and nitric oxide metabolite) are presented in Figure 1. As shown, the serum content of MDA, FRAP, TSH, and nitric oxide metabolite in asthma and control groups were not remarkably differentiable. DTX administration significantly reduced serum FRAP levels compared to the asthma mice (*p* < 0.05); however *NOE* administration showed no effect. Our analysis also indicated that both *NOE* and DTX had no significant effect on serum MDA, TSH, and nitric oxide metabolite levels in asthma groups.

### 3.2. Effects of *NOE* on BALF Oxidative Stress Markers

Our findings proved that the lung FRAP level was markedly enhanced in the *A* group in comparison with the *C* group (*p* < 0.05), while tissue nitric oxide metabolite content showed no significant changes (Figure 2). The treatment with *NOE* at a dose of 500 mg/kg and DTX at a dose of 2.5 mg/kg greatly reduced the tissue FRAP levels as compared to the *A* group merely (*p* < 0.05).

### 3.3. Antioxidant Enzymes Activity in Lung Tissue

As indicated in Figure 3, the activity of GPX enzyme is significantly reduced in the *A* group compared to the *C* group (*p* < 0.05). Most importantly, the GPX activity in rats treated with *NOE* was increased markedly in compared to the *A* group (*p* < 0.05). Our findings showed that the SOD activity was slightly decreased in the *A* group in comparison with the *C* group (*p* < 0.05), while *NOE* extract slightly increased it in comparison to *A* group (Figure 3).

### 3.4. Effects of *NOE* on Gene Expression and Protein Levels of Inflammatory Markers

The expression of *α*-SMA, IL-1, and TGF-*β*, as pro-inflammatory genes was significantly elevated in the lung tissue of *A* group in contrast to *C* rats (*p* ≤ 0.05) (Figures 4(b)–4(d)). Our results indicated that *NOE* and DTX at dosages of 500 mg/kg and 2.5 mg/kg, respectively, reduced the relative expression of *α*-SMA contrast to the asthma group (*p* < 0.05) (Figure 4(c)). The results further showed that *NOE* had no effect on TGF-*β* expression against the asthma mice, however DTX significantly reduced its level (*p* < 0.05) (Figure 4(d)). Moreover, measuring the TNF-*α* levels demonstrated no significant differences between experimental groups in the TNF-*α* level (Figure 4(a)). On the other hand, both DTX and *NOE* were able to reduce IL-1B levels compared to the asthma group but were not statistically significant.

As illustrated in Table 1, the expression of TNF-*α*, IL-10, and IL-6 genes in the asthma group showed no significant difference compared to the other groups.

### 3.5. Histological Experiments

The histopathological evaluation of lung tissue showed that the inflammatory cells in the asthma group is penetrated into the surrounding bronchial tissues leading to alveolar damage and terminal bronchial destruction, whereas this effect was not detected in the control group. In contrast, *NOE* was able to reduce inflammation and improve the morphological symptoms similar to DTX (Figure 5).

## 4. Discussion

Asthma is one of the most common chronic inflammatory disorders of the airways, characterized by airway hyper responsiveness and caused by infiltrative inflammatory cells and mucus hypersecretion [44]. Exposure of animals to OVA protein through the airways creates a pattern of airway inflammation that develops cellular and pathophysiological features similar to human asthma [45]. In the present study, a rat model of allergic asthma was developed in order to evaluate the effects of *NOE* on oxidative stress and inflammation markers.

Glucocorticoids are the most common anti-inflammatory drugs for the clinical treatment of asthma that can effectively suppress airway inflammation [46]. Therefore, we used dexamethasone as a positive control drug to compare the effectiveness of *NOE* with dexamethasone in reducing asthma.

One of the pathological factors associated with the onset and progression of asthma is oxidative stress [47]. During the process of developing asthma, inflammatory immune cells (neutrophils, eosinophils, monocytes, and macrophages) and epithelial cells produce ROS. By generation of ROS, higher content than the natural antioxidant capacity of the lungs, oxidative stress and cell damage occur [48]. Excessive oxidative stress has been reported to exacerbate sputum production and inflammation in the airways and damage respiratory epithelial cells [12]. Nitric oxide is a free radical and a highly reactive mediator that rapidly reacts with superoxide anions and consequently forms peroxide nitrite. Nitrite peroxide is a powerful oxidizer that can damage DNA, protein, and fat in biological membranes [23]. Our findings showed that the serum nitric oxide content in *A* rats receiving *NOE* was slightly decreased compared to the *A* animals. Furthermore, there was no significant difference about the TSH levels between all groups. Duration of the *NOE* application or the lower dose used in our study might be the rationale of the slight change in oxidative stress markers between the studied groups.

FRAP is a useful indicator of total antioxidant capacity that measures antioxidant components such as ascorbic acid, phenols, *β*-carotene, and uric acid [49]. Many studies showed diminished FRAP or total antioxidant capacity in asthma [50, 51]. Our findings also showed a significant decrease in FRAP levels in group *A* compared to group *C*.

To fight oxidative stress, lung and blood cells have several antioxidant defense systems, including enzymatic agents (SOD, CAT, and GPX) and nonenzymatic ones (vitamins E, C, and glutathione) [52]. The enzyme SOD plays a key role in the removal of ROS because it reduces superoxide (O_2_^‒^) to form hydrogen peroxide (H_2_O_2_). The CAT catalyzes the breakdown of H_2_O_2_ produced by SOD into water and oxygen, leading to protect the cell from the harmful effects of H_2_O_2_ [9]. In the present study, a slight reduction in SOD and a marked reduction in GPX activity were observed in *A* group compared to the *C* group. Many studies are in consistent to our results [41, 53]. Previously published data show that *NOE* consumption significantly increases the activity of SOD enzyme [54]. This study also confirmed that *NOE* had an effect on the GPX and SOD activity in the group *A* + *NOE* compared to group *A*. These findings increased the knowledge of the antioxidant effects of *NOE*, in which, the phenolic compounds stimulate GPX activity, thus reducing the free radical accumulation [55]. Therefore, it can be concluded that the *NOE* has a protective ability against oxidative stress for maintaining lung function. Based on the phenolic content of this plant previously reported, mainly flavonoids and phenolic acids [56], it can be hypothesized that those compounds may be the responsible compounds for this bioactivity.

In the pathogenesis viewpoint of asthma, oxidative stress is associated with inflammation and remodeling [57]. Inflammation of the airways is mainly caused by Th1 and Th2 cells, which secrets various cytokines. These cells also release more inflammatory and oxidative molecules that damage lung cells and tissue [10]. The activated Th2 cells release high level of cytokines, including IL-4, IL-5, and IL-13, leading to trigger AHR, induce mast cells, infiltrate eosinophils into the lungs, and subsequently increase mucus secretion [48]. Several studies reported that the expression of TNF-*α*, TGF-b, IL-1B, and *α*-SMA genes is significantly increased in OVA-induced asthma in animals, which is consistent with our findings [13, 58, 59].

Previous studies confirmed that the *NOE* reduces inflammatory responses by inhibiting the expression of TNF-*α*, IL-1*β*, and IL-6 [60, 61]. According to our experiments, the administration of *NOE* also decreased the expression of TNF-*α*, IL-1*β,* and *α*-SMA similarly to the DTX treatment group in asthmatic rats. Moreover, a significant effect on *α*-SMA levels was observed among the studied groups.

According to our findings in line with a study performed by other investigations [14, 41], there is a significant difference in the IL-10 expression between the asthma and control groups.

One of the most important profibrotic cytokines is transforming growth factor *β* (TGF-*β*), which is increased with oxidative stress. This cytokine is produced by cells including macrophages, epithelial cells, fibroblasts, and eosinophils [13]. Evidence has shown that TGF-*β* induces epithelial cell apoptosis, microvascular changes, fibroblast cell proliferation, and their differentiation into myofibroblasts during the development of subepithelial fibrosis. It also promotes airway remodeling by enhancing the proliferation, survival, and secretion of extracellular matrix (ECM) in airway smooth muscle cells (ASMCs), thereby thickening the airway wall [62, 63]; it is worth mentioning that based on Ji et al., the epithelial-mesenchymal transmission (EMT) can be induced by TGF-*β* [64]. EMT is the process by which an epithelial cell becomes a more mobile mesenchymal cell, resulting in increased specific markers of mesenchymal cells such as *α*-SMA and vimentin [63]. In the present study, treatment with the *NOE* similar to DTX treatment significantly reduced overexpression of the *α*-SMA gene in OVA-induced asthmatic rats; also the *NOE* had a noticeable effect on the expression of the inflammatory gene TGF-*β*. In one study, the antioxidant and anti-inflammatory properties of NOE were suggested to protect against bleomycin-induced pulmonary fibrosis in a rat model [65]. Accordingly, several studies have reported anti-inflammatory, antioxidant, and immune-regulating effects of the *NOE* [60, 61]. This ability is due to the biological active compounds, particularly phenolics, glucosinolates, and carotenoids present in the plant, whilst much evidence approved the ability of these phytoconstituents to inhibit the production or activation of the pro-inflammatory mediators, which lead to anti-inflammatory potencies [66]. Thus, the *NOE* may improve airway remodeling and suppress inflammatory responses by inhibiting the inflammatory marker *α*-SMA and/or regulating the oxidant-antioxidant system.

As abovementioned, the key pathological indicator of asthma, despite all the components or allergic mechanisms causing this disease, is inflammation of the airways. The histopathological findings of this study also showed that *NOE* has excellent anti-inflammatory effects, since it significantly reduced the airway inflammation and alveolar damage in asthma mice.

## 5. Conclusion

Generally, the results of the present study showed that the *NOE* significantly can suppress the inflammatory responses, airway regeneration, hypertrophy, and smooth muscle cell hyperplasia by inhibiting *α*-SMA production in the asthmatic rat model. Moreover, the extract of this plant could improve oxidative stress in the lungs of asthma rats by improving GPX activity. We conclude that the plant has limited effect on oxidative stress and moderate effect on lung inflammation. Then, further studies are needed to confirm the antioxidant and anti-inflammatory effects of the different doses of *NOE*.

## Figures and Tables

**Figure 1:** The effect of *NOE* on serum oxidative stress markers in OVA-induced rats. FRAP: ferric reducing antioxidant power; TSH: total thiol group; MDA: malondialdehyde; C: control; A: asthma; *NOE*: 500 mg hydroalcoholic extract of *Nasturtium officinale*; DTX: 2.5 mg dexamethasone. Data are expressed as mean ± SEM; ^*∗*^significant difference compared to the *C* group. #significant difference compared to the *A* group (*p* < 0.05).

**Figure 2:** The effect of *NOE* on the FRAP (a) and nitric oxide metabolite (b) levels in the bronchoalveolar lavage fluid (BALF) in OVA-induced rats. FRAP: ferric reducing antioxidant power; NO metabolite: nitric oxide metabolite; C control; A asthma; *NOE*: 500 mg hydroalcoholic extract of *Nasturtium officinale*; DTX: 2.5 mg dexamethasone. Data are expressed as mean ± SEM; ^*∗*^significant difference compared to the *C* group (*p* < 0.05), ^#^significant difference compared to the *A* group (*p* < 0.05).

**Figure 3:** The effect of *NOE* on the antioxidant enzymes activity of SOD (a) and GPX (b) in the lung tissue in ovalbumin-induced rats. SOD: superoxide dismutase; GPX: glutathione peroxidase. C: control; A: asthma; NOE: 500 mg hydroalcoholic extract of *Nasturtium officinale*; DTX: 2.5 mg dexamethasone. Data are expressed as mean ± SEM; ^*∗*^significant difference compared to the *C* group (*p* < 0.05), ^#^significant difference compared to the *A* group (*p* < 0.05).

**Figure 4:** The effect of *NOE* on the mRNA levels of TNF-*α*, IL-1, TGF-*β*, and *α*-SMA in ovalbumin-induced asthmatic rats. Data are expressed as mean ± SEM; ^*∗*^significant difference compared to the *C* group (*p* < 0.05), ^#^significant difference compared to the *A* group (*p* < 0.05). C: control; A: asthma; *NOE*: 500 mg hydroalcoholic extract of *Nasturtium officinale*; DTX: 2.5 mg dexamethasone.

**Figure 5:** The effects of NOE on histopathological changes in a rat model of OVA-induced asthma. (a) Photomicrograph of the lung stained with haematoxylin and eosin (10x); (a): control; (b) asthma; (c) control group treated with 500 mg/kg of *NOE*; (d) asthmatic group treated with 2.5 mg/kg of dexamethasone; (e) asthmatic group treated with 500 mg/kg of *NOE*.

**Table 1:** Effect of *NOE* on the cytokine markers in OVA-induced asthma rats.

Groups	TNF-*α* (pg/ml)	IL-10 (pg/ml)	IL-6 (pg/ml)
*C*	15.96 ± 2.36	7.31 ± 0.29	3.92 ± 0.50
*A*	30.56 ± 2.88	7.56 ± 0.23	3.67 ± 0.09
*NOE*	37.74 ± 2.10	7.53 ± 0.35	3.65 ± 0.47
*A* + *NOE*	20.81 ± 1.80	7.67 ± 0.55	3.82 ± 0.09
*A* + DTX	29.53 ± 7.13	8.51 ± 0.47	3.61 ± 0.86

Values presented as mean ± SEM. C: control; A: asthma; *NOE*: 500 mg hydroalcoholic extract of *Nasturtium officinale*; DTX: 2.5 mg dexamethasone. TNF-*α*: Tumor Necrosis Factor *α*; IL-10: Interleukin-10; IL-6: Interleukin-6. Data are expressed as mean ± SEM; ^*∗*^significant difference compared to the *C* group (*p* < 0.05), ^#^significant difference compared to the *A* group (*p* < 0.05).

## Data Availability

The data supporting the findings of this study are available within the article.

## Abbreviations

AHR: Airway hyper responsiveness
Th2: T helper 2
IL-4: Interleukins-4
IL-6: Interleukin-6
IL-10: Interleukin-10
IL-1*β*: Interleukin-1*β*
TNF-*α*: Tumor Necrosis Factor *α*
TGF-*β*: Transforming Growth Factor-*β*
*α*-SMA: Smooth muscle actin-*α*
ROS: Reactive oxygen species
RNS: Active nitrogen species
RSS: Active sulfur species
CAT: Catalase
SOD: Superoxide dismutase
MDA: Malondialdehyde
PCO: Protein carbonyl
TSH: Total thiol group
FRAP: Ferric reducing antioxidant power
*NOE*: *Nasturtium officinale* extract
DTX: Dexamethasone
AMSC: Airway smooth muscle cells.
